This article has been retracted.

# Clinical Effect of Suture Anchor and Double-Pulley Technique in the Treatment of Inferior Patellar Fracture

**DOI:** 10.1155/2021/4964195

**Published:** 2021-12-31

**Authors:** Hang Yu, Hui Dong, Binjia Ruan, Xiaohang Xu, Yongxiang Wang, Le Hu

**Affiliations:** ^1^Clinical Medical College of Yangzhou University, Yangzhou, China; ^2^Northern Jiangsu People's Hospital Affiliated to Yangzhou University, Yangzhou, China; ^3^The Yangzhou School of Clinical Medicine of Dalian Medical University, Yangzhou, China

## Abstract

**Objective:**

To evaluate the efficacy of suture anchor combined with double-pulley technique for subpatellar comminuted fractures compared with wire vertical suture and Krachow in the treatment of subpatellar fractures.

**Methods:**

Retrospectively selected 48 patients with subpatellar pole comminuted fracture admitted in our hospital from February 2013 to July 2019, 25 patients with double-pulley technique (group A), and 23 patients with vertical wire suture with Krachow suture. Patient age, gender, AT/OTA typing, injury mechanism, follow-up time, surgical time, bleeding volume, mean fracture healing time, and postoperative complications were recorded. The Insall-Salvati index immediately and 6 weeks after surgery. Bostman scores and knee activity were recorded at each follow-up, and month 12 was taken as the final result.

**Results:**

Time of surgery in group A (46.52 min) was significantly shorter than in group B (76.30 min). Intraoperative bleeding in group 15.1 ml, B, group 15.9 ml. Both incisions healed in stage I, averaging clinical healing of patella fracture within 10 weeks. There was no significant difference in mean Bostman score and knee activity at month 12 (group A: 28.4, 124.8°; group B: 28.1, 125.7°). There was no significant statistical difference in the Insall-Salvati index immediately or 6 weeks between the two groups. Group B patients had two wire fractures, fracture healing and the wire removed one year after surgery, and the remaining patients had no complications such as internal fixation loosening, fracture, delayed healing, or nonhealing of fracture.

**Conclusion:**

Compared with the treatment of subpatellar fracture with wire vertical suture and Krachow method, suture anchor with double-pulley technique has short operation time, reliable fixation, and less complications. Patients can have early functional exercise and good knee function recovery without secondary surgery. It can be considered as an alternative therapy for this fracture and deserves clinical adoption and promotion.

## 1. Introduction

The patella is the largest seed bone in the human body and is an important part of the knee extension device. Knee extension dysfunction due to patella fractures accounts for about 1% of all fractures [1]. The subpatellar pole, the extension of unarticular cartilage in the anterior patella cortex, is the attachment point of the patella ligament. The occurrence of fractures is often caused by indirect violence, accounting for 9%-22.4% of all patellar fractures [2]. And most of them are completely comminuted fractures, and the vertical length is generally less than 15 mm.

This comminuted avulsion fracture, often due to obvious displacement or combined extensor structural fracture, may cause the loss of continuity of the knee extension device and the loss of coordination of the patellar-femoral joint. If the treatment is not timely, it will reduce the quality of life and even eventually lead to lifelong disability. Therefore, there is a proposition of early surgical treatment, to realize the functional recovery of the femoral quadriceps extensor muscle and fracture anatomical reduction and parallel strong internal fixation, to provide conditions for early functional exercise.

In the past, subpatellar resection was used in the treatment of subpatellar fractures, but scholars have shown that subpatellar resection can lead to lower patellar displacement, causing patellar femoral dislocation and traumatic patellar femoral arthritis [3]. And the patient's subjective satisfaction rate was low, and the knee function recovery was poor. Therefore, the idea of preserving patella fragments as much as possible is increasingly acceptable to orthopedic surgeons in the treatment of subpatella fracture, and subpatella resection is used as a secondary option or revision surgery after failure of the implant. In recent years, in order to retain the internal fixation method of the lower patellar pole, there are common wire tension band, basket net steel plate fixation, etc. Wire vertical suture combined with Krachow suture legal is also an effective method for the treatment of subpatellar pole fracture [4], less complications and good recovery of knee function. Some scholars have also used suture anchor fixation for the treatment of subpatellar pole fractures [5]. It can not only retain the distal patella fragments but also maintain the normal patella height and can conduct early functional exercise, providing the conditions for good functional recovery. However, each method has its advantages and disadvantages, none of which is universal. Studies have been partially reported to compare the fracture internal fixation method with subpatella pole resection, but few have been reported on the efficacy contrast of different internal fixation methods.

Therefore, this retrospective study evaluated the clinical efficacy of suture anchor combined with double-pulley technique for subpatellar comminuted fractures and was legally compared with wire vertical suture combined with Krachow suture.

## 2. Patients and Methods

### 2.1. Retrospectively Selected 48 Patients with Subpatellar Polar Comminuted Fractures Admitted to Our Hospital from February 2013 to July 2019

It was divided into 25 cases of group A with wire anchor and double-pulley suture technique and 23 cases of group B with legal technology for vertical wire suture and Krachow suture. The inclusion criteria were as follows: age 18, complete medical records; physical examination indicates knee dysfunction; imaging diagnosis diagnosed subpatellar fracture; surgical time within 7 days after injury. The exclusion criteria were as follows: severe osteoporosis, diabetes; difficult walking difficulties or limited function before injury; previous history of knee surgery; previous history of metabolic disease and psychosis (Figure 1).

The study was approved by the Medical Ethics Committee and subject to its supervision. All patients and their families signed informed consent, and the study complies with the provisions of the Declaration of Helsinki (revised in 2013 in Brazil).

Demographic and clinical characteristics, including age, sex, AT/OTA typing, and injury mechanisms, were recorded.

### 2.2. Operative Techniques

#### 2.2.1. Group A

After successful anesthesia, the surgical incision of the median knee joint was used. After revealing the fracture end, the local hematoma and the joint cavity were removed. The lower angles of the proximal fracture block entered two 5.0 mm anchors 45°. The fracture of the fracture end was initially restored with the reduction clamp and repaired the torn patellar ligament that was stitched. The same color suture of the anchors on both sides was sutured to the patellar ligament of the lower patellar pole and fixed. The anchor tail hole served as the pulley to reverse pull the other end of the same color line, and alternately tightened, so that the broken end is firmly fixed. The other end of the monochromatic line was again sutured on the patellar ligament of the lower patellar pole, tied, and fixed, so that the four fixed knots were evenly dispersed in the lower patellar pole to complete the double-pulley fixation. The cut anchor line is stitched with 8 words through the upper and lower patellar ligament to strengthen fixation (the upper pole can also be bone tunnel for 8 words of enhanced fixation). C-type perspective: satisfactory fracture reduction, internal fixation, active knee, see satisfactory activity, the skin was stitched layer by layer (Figures 2 and 3).

#### 2.2.2. Group B

Standard anterior knee median incision, after the fracture end through the posterior edge of the proximal fracture surface, pointing to the anterior edge of the patellar, by 2~3 stainless steel wire through the hole using reset clamp pull tightening reset, absorption line using Krachow joint legal cross-lock edge continuous suture anterior patellar tissue and parapatellar ligament; C perspective: fracture reset satisfaction, internal fixtures, active knee joint, see its activity, internal fixation (Figure 4).

### 2.3. Postoperative Treatment

Antibiotics were routinely used to prevent the infection until one day after surgery. At 24 h after surgery, the patient began to guide the femoral quadriceps contraction, straight leg elevation, ankle dorsal extension, plantar flexion activity, and other functional exercises, to prevent deep vein thrombosis. Three days after surgery, CPM knee flexion and extension exercise was performed, and the amplitude of knee flexion gradually increased. Within 1 month after the operation, under the protection of the support, help double turned off of bed without incomplete load, bed passive flexion and extension exercise (flexion 90°). Support protection was removed within the 1-2 months after surgery, and the load bearing was gradually strengthened. Two months after surgery, knee clinical findings and X-ray tablets were regularly reviewed at 1, 2, 3, 6, and 12 months after surgery.

### 2.4. Observation Indicators

Indicators were assessed for patella height based on the immediate and 6 weeks postoperative Insall-Salvati index. The Bostman patella fracture functional score was recorded for each follow-up [6] and mean functional recovery after the knee joint, using the 12th-month follow-up results as the final functional outcome. Regular postoperative follow-up assessed fracture healing based on clinical presentation and X-ray examination, postoperative complications were observed, and knee range of motion (ROM) was recorded at the last follow-up.

### 2.5. Statistical Methods

The data were analyzed using SPSS19.0 software. Measurement data are expressed as mean standard deviation (M ± SD), *t*-test comparison between two groups. All the data accord with the normal distribution. Count data are described as frequency (%) and *χ*^2^ test between groups. *P* < 0.05 was statistically significant.

## 3. Results

### 3.1. Patient Data

In this retrospective study (Table 1), a total of 48 fractures met the inclusion criteria: 25 in group A used suture anchor with double-pulley technique, and 23 in group B had wire vertical suture with Krachow suture: gender (15 men in group A, 10 women in group A; 17 men in group B and 6 women, *P* > 0.05), mean age (53.4 years in group A; group B 54.7 years, *P* > 0.05), AO/OTA fracture typing (group A 18 A1, 7 C1.3; B 15 A1, 8 C1.3, *P* > 0.05), mean after injury to surgical time (2 days in group A; B 2.6 days, *P* > 0.05), injury mechanism (23 falls, 2 others; 22 group B, 1 other, *P* > 0.05), and mean follow-up time (group A 18 months; group B 16 months, *P* > 0.05).

### 3.2. Functional and Clinical Outcomes

Average operation time: group A (46.52 ± 6.43 min) is shorter than group B (76.3 ± 7.86 min). Mean bleeding volume: 15.1 ml in group A and 15.9 ml in group B, with no significant difference.

The Insall-Salvati index (IS) was defined as the ratio of the patellar tendon length (measured from the distal patellar to the tibia nodules) to the maximum length of the patella (from the distal to the proximal end of the patella) [7]. Immediately postoperative IS: A group (0.98 ± 0.07) and B group (0.97 ± 0.06). Six weeks after IS: A (0.98 ± 0.05) and B (0.97 ± 0.06).

At 12-month follow-up of Bostman score, there was no significant difference between group A Bostman score (28.36 ± 1.29) and knee activity (ROM) (124.76 ± 7.24°) and group B (28.13 ± 1.22, 125.74 ± 6.88°) (Figure 5).

### 3.3. Complications

The incision healed in the first phase, and the clinical healing of patella fracture reached within 10 weeks of both groups, and X-ray examination at 6 months after surgery indicated bone healing. During the follow-up period, all 48 patients had no deep infection, group B, the wire was removed one year after surgery, and the rest had no complications such as internal fixation loosening, fracture, delayed fracture healing, or nonhealing (Table 2).

## 4. Discussion

The integrity of the patella is important for maintaining static and dynamic stability of the knee and enhanced strength of the quadriceps. It is reported that patella surface compression stress increased dramatically when descending or descending bending the knee by 45 to 60°, with patella-femoral joint action up to 3200 N, approximately 4 to 5 times of the body weight [8]. Therefore, if to meet the requirements of early functional exercise, there must be a strong internal fixation. The subpatellar part without cartilage attachment in the distal patella is hidden in the patellar ligament and subpatellar fat pad and does not participate in the composition of the patellar and femoral joint. Therefore, the subpatellar extreme avulsion fracture belongs to the external joint fracture, and its characteristics are small, mostly comminuted, thin sheet, and coronal stratification. Also because it is close to the starting point of the patellar tendon, when the stress is concentrated during the joint activity, it is difficult to maintain the effective reduction and strong fixation, which is the difficulty in the surgical treatment of internal fixation. Therefore, various internal fixation methods have been continuously reported in recent years [9–11]. However, there is a question about what surgery is superior.

The traditional TBW (Tension Band Wiring) fixation method through the patellar and tibial nodules is prone to internal fixation fracture and low patella, which ultimately affects the knee function, and has been rarely used in clinical practice [9]. The Kirschner wire TBW fixation technique can convert the front tension in flexion of the knee joint into compressive stress between fracture blocks, which is widely used in large fractures [12]. But there are also complications that cannot be ignored, and the subcutaneous prominent Kirschner wire and twisted wire ends stimulate the soft tissue, and a rate of 22% surgical failure was reported by Smith et al. [13]. For subpatellar comminuted fracture, Kirschner wire cannot find the ideal position below the patella because of the size of the small fracture block, and it is difficult to obtain effective reduction and strong fixation, which requires gypsum fixation or support for a long time, which is not conducive to early functional rehabilitation exercise and weight bearing. Chang and Ji [14] used a hollow screw instead of a Kirschner wire to treat the subpatellar pole fracture; follow-up found a loss of knee flexion in 57° of patients.

The patella basket plate is a bilateral structure that integrates the distal patellar fragments at the lower edge into the patella ligament and holds four screws at the fracture breakend to provide a stable bone connection, maintain the normal patella height, and realize the early functional exercise and weight bearing after surgery. Biomechanical tests showed that the maximum load of the basket steel plates can reach (421.66 ± 45.90) N, which is significantly improved compared with other internal fixation methods [15]. However, this technical disadvantage lies in the possible cause of patellar ligament damage, and the large volume of the plate and the thin soft tissue layer in front of the patella, and endoplant irritation may occur when flexion of the knee joint. At the same time, the particularity of the steel plate makes it only used in some medical institutions.

Independent vertical wire technology, using Kirschner wire through the posterior edge of the proximal fracture surface, pointing to the anterior upper edge of the patella drilling, 2-3 wire perforation around the distal patella bone block, and then through the patella ligament to the front of the patella, operation is simple to tighten. Yang and Byun [16] reported using this technique to treat subpatellar fracture, with good biomechanical properties and a stronger load than the tension band wire (250 N), but different complications were found in 1/4 patients during follow-up. As the strength of the quadriceps tendon reached 316 N during the knee extension, the separate vertical wire fixation still has problems in the rapid maintenance of small broken bones, and the functional exercise needs to be carried out gradually under the protection of the postoperative braces. It has also been reported that separate vertical wire techniques were improved by increasing the Krachow seam legality along both sides of the patellar ligament to improve fixation strength [4].

In this study, we used the suture anchor to fix the full proximal fracture; the anchor tail line applied a double-pulley technique to completely wrap the distal fracture and used the cut anchor line as an “8” tension band through the upper and lower patellar ligament to protect and assist the ribbon anchor. Anchor line strength significantly exceeds the general suture; Sasaki et al. [17] by comparing the mechanical characteristics of the screws and the anchor lines, it is found that there is no obvious statistical difference in the strength of the two lines, thus ensuring the early functional exercise after the operation. Suture anchor and double-pulley technique are widely used in shoulder surgery, such as bone Bankart injury, remplissage repair of shoulder instability, rotator cuff injury, and SLAP injury [18, 19]. It can provide a repair effect in a large range as well as provide a stable internal fixation effect. Subpatellar fracture is a kind of ligament avulsion fracture; to this end, we apply the double-pulley technology to this fracture, with the following advantages: (1) Four stitches through the junction of the distal patella and the patellar ligament, most of the subpatellar fracture block is suspended and fixed, in a hammock-like arc. Thus, the pressure on the fracture end is strong and even, providing the possibility for early functional exercise. (2) The placement of 45° into the oblique inward makes the long axis of the anchor 90° from the tail end, resulting in stronger pull-out resistance. In Kadar et al. [5] of the 27 cases with the suture anchor to treat the subpatellar pole comminuted fracture, 3 (11.11%) had a failure of internal fixation. In their case, the anchor tail was subjected to suture tension with the anchor long axis of 0°, whereas in Aktay and Kowaleski [20], the biomechanical experiments showed that the pull of the anchor tail is 90° from the anchor long axis than 0°. This may explain the emergence of early internal fixation failure in the study by Kadar et al. (3) The four-way suture can form a tension balance through the anchor tail hole serving as the pulley, avoiding the knot tightness difference leading to a more concentrated stress on a tighter line. In Douglass et al. [21], the finding was the most common form of anchor fixation failure when the anchor was pulled out. In Robb et al. [22], it was also noted that when each anchor is tied individually during this internal fixation, one anchor is always pulled out first than the other anchor. This may be due to the difference in the tightness of each anchor suture at knots, when flexion of the knee, the tightest knot is first tightened, leaving most of the tension borne by this anchor. (4) Stitched the cut anchor line ring and fixed the TBW to make the patella fracture further firmly fixed, and the thread junction is buried under the soft tissue to avoid cutting and friction between the joint during movement.

In this study, we assessed patella height by conventional X-ray Insall-Salvati index measurement, and both high or low patella can lead to knee dysfunction. The two groups were fixed immediately and 6 weeks after surgery, suggesting that there was no significant patella height change in the process of fracture healing, providing a good anatomical foundation for knee function recovery. However, at the 12-month follow-up, there was no significant difference between Bostman score and knee activity and group B, and both surgical methods on the surface could achieve good surgical results. And with line anchor method treatment of subpatellar fracture that has a variety of advantages, not only simple operation, small trauma (incision is about 6 cm), operation time is significantly shorter than group B, and patients have no internal fixation loosening complications. In group B, two cases of wire fracture, although did not cause fracture displacement, but the patient requested surgery to remove for a year after surgery, increased the risk of secondary injury. In this study, the suture anchor adopts high and low double thread design, fixed stably in bone without removal, avoiding secondary operation; small volume and good tissue integration, completely drilling into bone without contact with soft tissue, minimizing rejection, and allowing patients to undergo MRI examination.

The anchor fixation of the joint double-pulley technology requires two anchors as the fulcrum of the whole fixation system and depends on the integrity of the proximal fracture block. If there is also a comminuted fracture of the proximal fracture block, this method is not applicable and may cause anchor loss. Similarly, this fixation should be used with caution in patients with severe osteoporosis.

## 5. Conclusion

Compared with the legality of wire vertical suture and Krachow suture, suture anchor combined with double-pulley technique has a good treatment of subpatellar comminuted fracture reduction effect, reliable fixation, and few complications, and patients can have early function exercise and good knee function recovery after surgery, which is worthy of clinical adoption and promotion. However, this study was a retrospective study with a small sample size and patients were not randomized into two treatment groups. And some patients have a short follow-up time, and further large sample and long-term follow-up studies are needed.

## Figures and Tables

**Figure 1:** Preoperative knee radiographs. A female patient, 66 years old, was admitted to the hospital with a fall resulting in swelling of the right knee with limitation of movement, and a right knee X-ray in front and side view and 3D CT showed an inferior patella fracture with significant displacement.

**Figure 2:** Group A intraoperative. The anchors of the two anchors were sutured to the patellar ligament of the lower patellar pole and fixed (left). The anchor tail hole as the pulley to reverse pull the other end of the same color line and the other end of the monochromatic line was again sutured on the patellar ligament of the lower patellar pole, so that the four fixed knots were evenly dispersed in the lower patellar pole (right).

**Figure 3:** Postoperative X-ray front and side view (group A). Anchor sutures. Anchor nail in place and subpatellar pole repositioning with no significant displacement.

**Figure 4:** Postoperative X-ray front and side view (group B). Wire vertical suture and Krachow. Fracture repositioned and internal fixation in place.

**Figure 5:** Postoperative review of knee mobility. At 12-month follow-up, the patient's knee mobility was nearly 0-125°.

**Table 1:** Patient data.

Characteristic	Group double-pulley (A)	Group Krachow (B)	*P* value
Gender (example number, (%))			
Male	15 (60%)	17 (73.9%)	>0.05
Female	10 (40%)	6 (26.1%)	>0.05
Age (age)	53.4 ± 8.6	54.7 ± 8.1	>0.05
AO/OTA typing			
A1	18 (72%)	15 (65.2%)	>0.05
C1.3	7 (28%)	8 (34.8%)	>0.05
Mechanism of injury			
Fall and hurt oneself	23	22	>0.05
Other	2^1,2^	1^1^	>0.05
Injury to operation time (day)	0.82 ± 1.16	0.62 ± 1.18	>0.05
Follow-up time (month)	18.16 ± 5.15	16.74 ± 4.29	>0.05

^1^Traffic road. ^2^The height fell and hurt.

**Table 2:** Clinical results.

Characteristic	Group double-pulley (A)	Group Krachow (B)	*P* value
Operation time	46.52 ± 6.43	76.30 ± 7.86	<0.05
Amount of bleeding	15.16 ± 4.03	15.86 ± 3.89	>0.05
The Insall-Salvati index			
Immediately after surgery	0.98 ± 0.07	0.97 ± 0.06	>0.05
Six weeks after surgery	0.98 ± 0.05	0.97 ± 0.06	>0.05
Bostman score	28.36 ± 1.29	28.13 ± 1.22	>0.05
Knee joint mobility (R OM)	124.76 ± 7.24°	125.74 ± 6.88°	>0.05
Complication	0	2	<0.05

## Data Availability

The data used to support the findings of this study are available from the corresponding author upon request.
